The article "MRI Evaluation of Indomethacin Suppositories in the Prevention of Complications of Pancreatitis and Hyperamylasemia after Choledocholithiasis ERCP Based on Image Denoising Algorithm" was published in 2022. Journal: Comput Math Methods Med.

# MRI Evaluation of Indomethacin Suppositories in the Prevention of Complications of Pancreatitis and Hyperamylasemia after Choledocholithiasis ERCP Based on Image Denoising Algorithm

**DOI:** 10.1155/2022/4805185

**Published:** 2022-08-23

**Authors:** Fusheng Gao, Chuan Zhang, Yue Feng, Yutao Zhan

**Affiliations:** Department of Gastroenterology, Beijing Tongren Hospital, Capital Medical University, Beijing 100176, China

## Abstract

**Objective:**

To explore the value of MRI evaluation of indomethacin suppositories in the prevention of pancreatitis and hyperamylasemia in patients with common bile duct calculi after endoscopic retrograde cholangiopancreatography (ERCP) based on image denoising algorithm.

**Methods:**

A retrospective analysis in August 2020 to December 2021. Because of the common bile duct calculi hospitalized parallel ERCP operation, 89 cases of patients, according to the different postoperative treatments, were divided into group A (*n* = 44) and group B (*n* = 45), in which A set of separate application inhibits the pancreatic enzyme secretion after surgery drug treatment, and B group on the basis of group A linked with indole beauty Xinshuan treatment. The incidence of postoperative pancreatitis and hyperamylasemia was compared between the two groups. The levels of serum amylase were compared between the two groups. Patients in group B were diagnosed with pancreatitis by conventional MRI and MRI with denoising algorithm, respectively, and the imaging characteristics and diagnosis rate differences of the two methods were observed. ROC curve was drawn to evaluate the diagnostic efficacy of MRI denoising algorithm for postoperative pancreatitis and serum amylase level detection for hyperamylasemia.

**Results:**

The incidence of postoperative pancreatitis and hyperamylasemia in group B was significantly lower than that in group A (*P* < 0.05). There were 6 cases of postoperative pancreatitis in group B, 2 cases (33.33%) were diagnosed by conventional MRI, and 5 cases (83.33%) were diagnosed by MRI based on denoising algorithm. Although there was no significant difference in diagnosis rate between the two methods, the number of cases of pancreatitis diagnosed by MRI based on denoising algorithm was slightly higher than that by conventional MRI. Compared with conventional MRI images, MRI images with denoising algorithm showed that the number of cases with pancreatic swelling, the number of cases with pancreatic duct/bile duct dilation, and the number of cases with abdominal effusion were all high (all *P* < 0.05). ROC results showed that the area under the curve of MRI with denoising algorithm for the diagnosis of postoperative pancreatitis was 0.855, and the sensitivity was 89.40%. The specificity was 83.20%, and the area under the curve of serum amylase for postoperative hyperamylasemia was 0.893, the sensitivity was 89.80%, and the specificity was 85.20%, all of which had high diagnostic efficacy.

The article "MRI Evaluation of Indomethacin Suppositories in the Prevention of Complications of Pancreatitis and Hyperamylasemia after Choledocholithiasis ERCP Based on Image Denoising Algorithm" was published in 2022. Journal: Comput Math Methods Med.

**Conclusion:**

MRI results of denoising algorithm suggest that indomethacin suppositories can effectively reduce the incidence of postoperative pancreatitis and hyperamylasemia after ERCP, which is worthy of clinical application.

## 1. Introduction

As the most common disease in the digestive system, choledocholithiasis can be divided into primary and secondary stones according to different sources, and the incidence of choledocholithiasis has been increasing year by year with the development of social economy and the change of dietary structure [1]. At present, there has not been a unified conclusion on the causes of choledocholithiasis in clinical practice, and most studies show that it is closely related to age, hypothyroidism, gastrointestinal dysfunction, and Oddi sphincter dysfunction [2]. The main clinical symptoms of such diseases are abdominal pain, jaundice, chills, and high fever. If medical treatment is not timely, it is highly likely to cause secondary infection and cholangitis and then induce systemic infection, endangering the life and health of patients [3]. Endoscopic retrograde cholangiopancreatography (ERCP) is widely used in the diagnosis and treatment of clinical hepatobiliary and pancreatic diseases and also has high clinical efficacy in the treatment of choledocholithiasis. However, some scholars have pointed out that pancreatitis and hyperamylasemia caused by ERCP are inevitable in the long-term clinical application process. Therefore, it is of great significance to seek a treatment that can effectively reduce postoperative complications of ERCP to improve the prognosis of patients with choledocholithiasis [4, 5]. In the past clinical practice, doctors usually give patients indomethacin before surgery to reduce the incidence of postoperative complications, but the drug delivery way will be complicated by gastric mucosal injury after surgery, so this study by adopting indomethacin suppositories in anus to medicine way, the effect of postoperative complications in patients with lower ERCP was observed, and the denoising algorithm of magnetic resonance imaging (MRI) to evaluate the specific efficacy is presented as the following reports [6].

## 2. General Information and Methods

### 2.1. General Information

A retrospective analysis was performed on 89 patients admitted for choledocholithiasis and undergoing ERCP from August 2020 to December 2021, who were divided into group A (*n* = 44) and group B (*n* = 45) according to different postoperative treatment methods. The baseline data of the two groups are shown in Table 1, which were comparable (*P* > 0.05). All the patients included in the study signed informed consent before surgery. In addition, we have the right to know the treatment and detection methods adopted in this study. The clinical data and general information obtained in this study are kept confidential and will not be used for other purposes. This study was approved by the Ethics Committee.

The article "MRI Evaluation of Indomethacin Suppositories in the Prevention of Complications of Pancreatitis and Hyperamylasemia after Choledocholithiasis ERCP Based on Image Denoising Algorithm" was published in 2022. Journal: Comput Math Methods Med.

Inclusion criteria are as follows: (1) it met the clinical diagnostic criteria for common bile duct calculi [7]. These include biliary colic caused by bile duct obstruction, cholangitis caused by secondary bacterial infection, abdominal pain, jaundice, chills, and high fever; (2) signed the informed consent before surgery; (3) ERCP operation was used in all cases; and (4) complete clinical data and general information.

Exclusion criteria are as follows: (1) accompanied by mental diseases, (2) intolerant to surgery, (3) congenital immune dysfunction or coagulation disorder, (4) deviation of study results caused by private use of other drugs during treatment; and (5) people who have allergic contraindications to the drugs used in the treatment process.

### 2.2. Methods

#### 2.2.1. MRI Detection of Image Denoising Algorithm

MRI images of patients in group B were detected by conventional MRI and denoising algorithm, respectively. The operation contents of each detection are as follows:

MRI was examined using a superconducting magnetic resonance imaging scanner (purchased from GE Corporation; Model: Discovery 750); before the test, it is required to fast and forbid water for 12 h and hold your breath for 20 seconds. It is forbidden to wear any metal jewelry during the test. The abdominal coil was a 32-channel phased array, and the cross-sectional unit first fired a single fast spin echo T2WI scan sequence. The scan sequence was set as layer thickness (5 mm), matrix (320 × 256), layer spacing (1 mm), field of vision (340 × 340) mm, and repeat time (TR)/echo time (TE) 4500/120 ms. The scan sequence was set as layer thickness (5 mm), matrix (224 × 180), layer spacing (1 mm), field of vision (340 × 340) mm, and TR/TE 2500/110 ms. T1WI fat suppression sequence scanning was performed by rapid volumetric imaging of liver (TR/TE3.6/1.7 ms), layer thickness (5 mm), matrix (224 × 180), and field of vision (360 × 360) mm. Contrast agent was injected at a rate of 2~3 mL/s with a special dual-tube high-pressure syringe for MR, and 20 mL 0.9% sodium chloride solution was injected with the same flow rate group. Continuous scanning was performed for 40 times.

The article "MRI Evaluation of Indomethacin Suppositories in the Prevention of Complications of Pancreatitis and Hyperamylasemia after Choledocholithiasis ERCP Based on Image Denoising Algorithm" was published in 2022. Journal: Comput Math Methods Med.

The denoising model is constructed as follows. The MRI image obtained above is given a noisy MRI *Y*, and the image is obtained by partitioning block set *RY* = (*R*_1_*Y*, *R*_2_*Y*, ⋯.., *R*_*m*_*Y*), *RY* was divided into class *K* by GMM prior, and *R*_*K*_*Y* = [*R*_*K*1_, *R*_*K*2_, ⋯, *R*_*Kd*(*k*)_] was used to represent the moment blocks composed of all image blocks in class *K* and decomposed according to the formula ${\bar{R}}_{K}Y=Z_{K}+N_{X}$ (*ZK* and *NX* are low-rank matrices and noise matrices, respectively). Assuming that the noise at each pixel in the image is independently distributed, the value of *Z*_*K*_ can be obtained according to the following formula:

(1) $$\begin{array}{c} E\left(Z_{K}\right)=\tau \left\|Z_{K}\right\|.+{\left.\frac{1}{\sigma^{2}}{\bar{R}}_{k}Y-Z_{K}\right\|}_{F}^{2}, \end{array}$$

where *τ* is constant and *σ* is noise standard deviation. By summarizing the given noisy MRI *Y*, the denoised MRI *X* is reconstructed by the following formula:

(2) $$\begin{array}{c} \;\left(\hat{X},\hat{C},\left\{{\hat{Z}}_{K}\right\}\right)=\underset{X,C,\left\{Z_{K}\right\}}{\text{argmin}}\frac{\lambda }{\sigma^{2}}{\left\|Y-X\right\|}_{2}^{2}-\log p\left(RY,C\left|\Theta \right.\right)+\overset{K}{\underset{k=1}{\sum }}E\left(Z_{K}\right), \end{array}$$

where *λ* is a constant and  *σ* is the noise standard deviation, and the clustering visualization result under GMM prior in Figure 1 can be obtained. The result shows that with the increase of the number of cycles, the MRI image can be effectively close to the denoised MRI.

#### 2.2.2. Serum Amylase Detection

5 ml of fasting venous blood was extracted from the two groups in the morning and put into a centrifuge with centrifuge parameters of 3500 r/min and centrifuge radius of 13.5 cm. After centrifugation for 10 min, the blood was placed under low temperature to be tested. A dry chemical automatic biochemical analyzer was used (purchased from Johnson & Johnson, USA, Model: VITROS950), serum amylase level was detected by dry biochemical assay, and the normal value was <200 U/L.

#### 2.2.3. Treatment Methods

ERCP was performed by the same team in both groups. Diazepam 10 mg (manufacturer: Dubeite Pharmaceutical Co., Ltd., National Drug Approval H41020631, specification: 10 mg), scopolamine 20 mg (purchased from Henan Furen Huaiqingtang Pharmaceutical Co., Ltd., National Drug Approval H19994038, specification: 1 ml : 0.3 mg), and 0.3 mg octreotide were given to group A (purchased from Beijing Baiao Pharmaceutical Co., Ltd., National Drug Approval H20061309, specification: 1 ml : 0.1 mg), and continuous intravenous infusion was performed 6 h before surgery. Group B was combined with indomethacin suppository (purchased from Beijing Shuangji Pharmaceutical Co., Ltd., H11021391, specifications: 100 mg) on the basis of group A, and anal plug was performed 30 min before surgery. Both groups were given the same anti-infection operation after surgery and observed.

The article "MRI Evaluation of Indomethacin Suppositories in the Prevention of Complications of Pancreatitis and Hyperamylasemia after Choledocholithiasis ERCP Based on Image Denoising Algorithm" was published in 2022. Journal: Comput Math Methods Med.

#### 2.2.4. Diagnostic Criteria for Pancreatitis

Diagnostic criteria for acute pancreatitis was divided into three, specified as follows: first, the pain symptoms: pancreatitis, typical pain symptoms are severe, mainly located in the upper abdomen, generally will appear early in the abdomen to the left or on the entire abdominal pain, have serious pain even when it appears late in the abdomen, all of them, and will start from light to heavy. Second, changes in blood amylase: the value of blood amylase exceeds more than three times the normal value, the general blood amylase will increase in the initial 2-12 hours of acute pancreatitis attack, and if the increase is more than three times, it represents the positive diagnostic criteria. Third, imaging examination: this includes B ultrasound, CT, and other examinations; there are typical changes in peripheral necrosis of pancreatitis, which suggest acute pancreatitis. If two of the three criteria are positive, the condition is often diagnosed as acute pancreatitis.

### 2.3. Statistical Treatment

The SPSS 25.0 statistical software was used for data analysis. (1) Measurement data: If the data followed normal distribution and homogeneity of variance after normality test, it was represented by mean ± standard deviation. Paired sample *t* was used for intragroup test, and variance comparison was used between groups. (2) Count data: Descriptive statistical analysis was conducted by percentage, and *χ*^2^ test was performed. (3) ROC curve was drawn to evaluate the diagnostic efficacy of MRI denoising algorithm for postoperative pancreatitis and serum amylase level detection for hyperamylasemia. All the above data showed significant differences with *P* < 0.05.

## 3. Results

### 3.1. To Compare the Incidence of Postoperative Pancreatitis and Hyperamylasemia

The incidence of postoperative pancreatitis and hyperamylasemia in group B was significantly lower than that in group A (*P* < 0.05), as shown in Table 2.

### 3.2. Serum Amylase Levels Were Compared after Operation

The postoperative serum amylase level in group B was significantly lower than that in group A (*P* < 0.05), as shown in Table 3.

### 3.3. Comparison of Imaging Characteristics and Diagnosis Rates of Different MRI Detection Methods

There were 6 cases of postoperative pancreatitis in group B, 2 cases (33.33%) were detected by conventional MRI, and 5 cases (83.33%) were detected by MRI based on denoising algorithm. Although there was no significant difference in diagnosis rates between the two methods, the number of cases of pancreatitis detected by MRI based on denoising algorithm was slightly higher than that of conventional MRI. The differences in imaging characteristics of the two detection methods are shown in Table 4 and Figures 2 and 3. The results showed that compared with conventional MRI images, MRI images with denoising algorithm showed higher cases of pancreatic swelling, dilatation of pancreatic duct/bile duct, and combined with abdominal effusion (all *P* < 0.05).

The article "MRI Evaluation of Indomethacin Suppositories in the Prevention of Complications of Pancreatitis and Hyperamylasemia after Choledocholithiasis ERCP Based on Image Denoising Algorithm" was published in 2022. Journal: Comput Math Methods Med.

### 3.4. ROC Evaluation of MRI Diagnostic Value of Denoising Algorithm for Postoperative Pancreatitis

ROC curve (Figure 4) showed that denoised MRI had high diagnostic value for postoperative pancreatitis in patients with ERCP, and its area under the curve was significantly higher than that of conventional MRI. The diagnostic efficacy is shown in Table 5.

### 3.5. ROC Evaluation of Serum Amylase Detection in the Diagnosis of Postoperative Hyperamylasemia

ROC curve (Figure 5) showed that serum amylase had high diagnostic value in patients with hyperamylasemia after ERCP surgery, with a line area of 0.893 and high specificity and sensitivity. The diagnostic efficacy is shown in Table 6.

## 4. Discussion

As an important way of clinical diagnosis and treatment of biliopancreatic diseases, ERCP has become the preferred treatment for choledocholithiasis in the application history of more than 30 years. However, some scholars pointed out that postoperative complications of ERCP are still unavoidable at present, especially the common postoperative acute pancreatitis and hyperamylasemia. Therefore, it is of great significance to seek a way to effectively reduce postoperative complications of ERCP for such patients [8, 9]. Indomethacin suppositories, as a commonly used drug in ERCP, can reduce the incidence of postoperative pancreatitis and hyperamylasemia to a certain extent, but its gastrointestinal irritation may cause complications related to the digestive system [10]. Therefore, indomethacin suppositories were adopted in this study to avoid gastrointestinal irritation by anal insertion, and its influence on reducing the incidence of postoperative complications in ERCP patients was further observed. In addition, MRI imaging technology with denoising algorithm was used to further evaluate the clinical efficacy of the drug. Lay a theoretical foundation for improving the prognosis of patients with choledocholithiasis in clinic [11].

The results of this study showed that indomethacin suppositories were given to patients 30 min before surgery, which could significantly reduce the incidence of postoperative pancreatitis and hyperamylasemia, and the serum amylase expression in group B was significantly lower than that in group A (*P* < 0.05). To analyze the mechanism of action of these results may after the author thinks that due to trigger factors including intraoperative ERCP postoperative pancreatitis mechanical injury, infection, and related inflammation, so by taking a certain means to control inflammation factor to reduce inflammation plays an important role to reduce the incidence of postoperative ERCP pancreatitis [12]. Indomethacin suppositories, as a kind of nonsteroidal anti-inflammatory drugs (NSAIDs), through the rectum can inhibit PLA2 activity after the treatment and prevent neutrophil leads to the organization, further blocking mediated by phospholipase A2 a large release of proinflammatory factor, secretion, thereby reducing the body's inflammatory response and reduce the incidence of postoperative pancreatitis and high blood amylase [13]. Li et al. [14] also showed in the study that indomethacin suppositories, as a phospholipase A2 antagonist, can inhibit prostaglandin activity and regulate inflammatory factor-related transmitters such as platelet active factor and interleukin, which can block the expression activity of inflammatory cytokines in the early stage of inflammation so as to prevent the inflammatory waterfall reaction. Thus, it can reduce postoperative complications, which is consistent with the results of this study.

The article "MRI Evaluation of Indomethacin Suppositories in the Prevention of Complications of Pancreatitis and Hyperamylasemia after Choledocholithiasis ERCP Based on Image Denoising Algorithm" was published in 2022. Journal: Comput Math Methods Med.

In addition, MRI with denoising algorithm was used to further evaluate the specific efficacy of indomethacin suppositories. Since ordinary MRI is prone to noise pollution in the imaging process, there is a certain deviation in the evaluation of image results. Therefore, in order to obtain high-quality MRI images and evaluate the specific efficacy of indomethacin suppositories, in this study, GMM was used to conduct the prior of noise images and low-rank rectangular decomposition algorithm was used for denoising [15, 16]. After denoising processing, MRI images showed A group of patients with postoperative swelling; the number of cases of pancreas and pancreatic duct/bile duct expansion in the number of cases occurred, and merger of peritoneal effusion was significantly higher than that of group B; prompt after denoising MRI images can be various and multidimensional imaging; high-resolution display of pancreatic necrosis area, at the same time, is under the condition of noninvasive assessment of the change of the bile duct, which clearly shows whether there are complications in local areas [17]. In addition, the ROC curve showed that MRI images of the denoising algorithm had a high diagnostic efficiency for the diagnosis of acute pancreatitis after ERCP, with an area of 0.855 under the curve. Meanwhile, timely detection of serum amylase level in patients after ERCP could also predict the occurrence of hyperamylasemia and take relevant measures to prevent the occurrence of adverse prognosis in time [18].

The article "MRI Evaluation of Indomethacin Suppositories in the Prevention of Complications of Pancreatitis and Hyperamylasemia after Choledocholithiasis ERCP Based on Image Denoising Algorithm" was published in 2022. Journal: Comput Math Methods Med.

To sum up, indomethacin suppositories can significantly reduce the common bile duct calculi patient pancreatitis and the probability of high blood amylase after ERCP, and the denoising algorithm of postoperative pancreatic imaging features of MRI image display of group B was significantly better than that of group A, further illustrating indomethacin suppositories for improving the prognosis of patients with common bile duct calculi ERCP postoperative outcome have high clinical curative effect. However, due to the small sample size of this study, the results lack a certain degree of rigor. Therefore, the sample size can be expanded in the next study, and cluster analysis of the results can be carried out to further observe the improvement effect of indomethacin suppositories on postoperative complications of ERCP, so as to make the results more rigorous and accurate.

## Figures and Tables

**Figure 1:** Denoising image processing process. Note: (a) the obtained original noise image, (b) the clustering result after 10 cycles, and (c) the clustering result of denoised MRI.

**Figure 2:** Conventional MRI image. Note: (a, b) conventional MRI images, showing poorly defined boundaries of the pancreas.

**Figure 3:** Denoised MRI image of a postoperative pancreatitis patient. Note: the figure shows denoised MRI images of patients with postoperative pancreatitis, in which the arrow in (a) shows large nonenhanced manifestations of pancreas and surrounding area, and the arrow in (b) shows T1WI image, with high shadow at the site indicated by the arrow, indicating the possibility of bleeding.

**Figure 4:** ROC image of pancreatitis on denoised MRI.

**Figure 5:** Diagnostic value of serum amylase in postoperative hyperamylasemia.

**Table 1:** The baseline data (*n*(%))/(*x̅*±*s*).

	A group (*n* = 44)	B group (*n* = 45)	*t*/*χ*^2^	*P*
Age (years)	46.55 ± 5.31	45.98 ± 4.86	0.527	0.610
Gender			0.096	0.756
Man	21 (47.73%)	20 (44.44%)		
Woman	23 (52.27%)	25 (55.56%)		
BMI (kg/m^2^)	23.21 ± 1.89	23.18 ± 2.05	0.080	0.937
Level of education			0.087	0.541
Primary and below	9 (20.45%)	11 (24.44%)		
Junior to senior high	23 (52.27%)	20 (44.44%)		
University and above	12 (27.27%)	14 (31.11%)		

**Table 2:** Comparison of postoperative complications (*n*(%)).

Group	*n*	Hyperamylasemia	Mild pancreatitis	Moderate pancreatitis
A group	44	10 (22.73%)	9 (20.45%)	5 (11.36%)
B group	45	3 (6.67%)	4 (8.89%)	2 (4.44%)
*χ* ^2^		4.601	4.363	
*P*		0.032	0.037	

The article "MRI Evaluation of Indomethacin Suppositories in the Prevention of Complications of Pancreatitis and Hyperamylasemia after Choledocholithiasis ERCP Based on Image Denoising Algorithm" was published in 2022. Journal: Comput Math Methods Med.

**Table 3:** Comparison of serum amylase levels (*x̅*±*s*).

Group	*n*	Amylase (U/L)
A group	44	298.35 ± 13.19
B group	45	256.42 ± 12.05
*t*		15.658
*P*		<0.001

**Table 4:** MRI observation of pancreatic imaging characteristics with denoising algorithm (*n*(%)).

	Conventional MRI detection (*n* = 45)	MRI detection with denoising algorithm (*n* = 45)	*t*/*χ*^2^	*P*
The pancreas swelling			4.686	0.030
Y	14 (31.11%)	5 (11.11%)		
N	31 (68.89%)	40 (88.89%)		
Whether the pancreatic duct/bile duct is dilated			3.902	0.048
Y	17 (37.78%)	8 (17.78%)		
N	28 (62.22%)	37 (82.22%)		
Combined with peritoneal effusion			5.099	0.024
Y	13 (28.89%)	4 (8.89%)		
N	32 (71.11%)	41 (91.11%)		
T1WI signal			4.994	0.025
High	21 (46.67%)	31 (68.89%)		
Low	24 (53.33%)	14 (31.11%)		
T2WI signal			5.756	0.016
High	19 (42.22%)	8 (17.78%)		
Low	26 (57.78%)	37 (82.22%)		

**Table 5:** Diagnostic efficacy of denoised MRI.

	95% CI	Sensitivity (%)	Specificity (%)	AUC	Cutoff value
Denoising MRI	0.774~0.925	89.40%	83.20%	0.855	--
Conventional MRI	0.704~0.873	84.50%	78.60%	0.787	--

**Table 6:** Diagnostic efficacy of serum amylase.

	95% CI	Sensitivity (%)	Specificity (%)	AUC	Cutoff value
Amylase	0.773~0.912	89.80%	85.20%	0.893	201.31 U/L

## Data Availability

The dataset used in this paper are available from the corresponding author upon request.
